# Long noncoding RNA ILF3-AS1 promotes cell proliferation, migration, and invasion via negatively regulating miR-200b/a/429 in melanoma

**DOI:** 10.1042/BSR20171031

**Published:** 2017-11-06

**Authors:** Xiangjun Chen, Sha Liu, Xiaochun Zhao, Xiao Ma, Guozhen Gao, Li Yu, Dexiong Yan, Hao Dong, Weijing Sun

**Affiliations:** 1 Department of Burn and Plastic Surgery, The 253rd Hospital of PLA, Hohhot, Inner Mongolia 010051, China; 2 Intensive Care Unit, The 253rd Hospital of PLA, Hohhot, Inner Mongolia 010051, China; 3 Department of General Surgery, The 253rd Hospital of PLA, Hohhot, Inner Mongolia 010051, China

**Keywords:** cell migration, EZH2, long noncoding RNA, melanoma, miR-200s, proliferation

## Abstract

Melanoma is the most malignant skin cancer, which account for most of skin-cancer-related deaths. Long noncoding RNA (lncRNA) is a class of noncoding RNAs with crucial roles in many cancers. However, the roles of lncRNAs in melanoma have not been well studied. In the present study, using public available data and clinical tissues samples, we found that lncRNA ILF3-AS1 is up-regulated in melanoma tissues and cell lines, and correlated with poor prognosis of melanoma patients. Functional experiments showed that knockdown of ILF3-AS1 inhibits melanoma cell proliferation, migration, and invasion. Mechanistically, we found that ILF3-AS1 interacts with EZH2, promotes the binding of EZH2 to the *miR-200b/a/429* promoter, and represses miR-200b/a/429 expression. The expression of ILF3-AS1 is negatively correlated with that of miR-200b/a/429 in melanoma tissues. Moreover, inhibition of miR-200b/a/429 abrogates the biological roles of ILF3-AS1 knockdown on melanoma cell proliferation, migration, and invasion. In conclusion, these results demonstrate that melanoma-upregulated lncRNA ILF3-AS1 promotes cell proliferation, migration, and invasion via negatively regulating miR-200b/a/429, and imply that ILF3-AS1 may be a potential prognostic biomarker and therapeutic target for melanoma.

## Introduction

Derived from malignant transformation of melanocytes, melanoma is the most aggressive skin cancer, which accounts for 75% of all skin-cancer-related deaths [1,2]. The incidence of melanoma is steadily rising, but the prognosis of melanoma patients is still very poor, especially for those with distant metastasis and at late stages of melanoma [3]. Despite recent advances in molecularly targeted therapy and immunotherapy, melanoma rapidly develops resistance to these therapies [4–6]. Therefore, revealing the molecular mechanisms underlying melanoma progression and designing rational therapeutic interventions are critical for the management of melanoma [7].

With great advances of high-throughput RNA sequencing technology, many reports have shown that most of human transcriptome could be classified as long noncoding RNAs (lncRNAs) [8,9]. LncRNA is a class of noncoding RNA with more than 200 nucleotides in length [10,11]. Accumulating evidence demonstrate that lncRNAs play important roles in tissue physiology and diseases processes, including cancers [12–16]. Many lncRNAs show aberrant expressions in a variety of cancers, and some dysregulated lncRNAs function as oncogenes or tumor suppressors in particular conditions [17–19]. However, the functions and action mechanisms of lncRNAs in melanoma are still poorly understood [20].

Another important group of noncoding RNAs is the microRNAs (miRNAs), which are typically 20–25 nucleotides in length [21]. The well-studied noncoding RNAs also have important roles and are frequently dysregulated in cancers [22–25]. The miR-200 family (miR-200s) is well known to function as tumor suppressors via inhibiting tumorigenesis and progression in many cancers [26,27]. miR-200s contains two clusters, with miR-200b, miR-200a, and miR-429 as the first cluster, and miR-200c and miR-141 as the second cluster. miR-200s are frequently dysregulated in many cancers, including melanoma [28,29]. But the factors contributing to the dysregulation of miR-200s in melanoma are still unknown.

In the present study, using a previously reported RNA sequencing results of melanoma [30], we found that lncRNA ILF3-AS1 (XLOC_013222, Refseq NR_024333.1) is up-regulated in melanoma. We further detected ILF3-AS1 expression in public available database and our own cohort of melanomas. Moreover, the biological roles and action mechanisms of ILF3-AS1 in melanoma are also investigated.

## Materials and methods

### Tissues samples

A total of 37 benign nevi, 60 primary melanomas, 25 metastatic melanomas, 13 breast tissues, 12 breast cancer tissues, 8 metastatic breast cancer tissues, 11 lung tissues, 9 non-small cell lung cancer (NSCLC) tissues, and 6 metastatic NSCLC tissues were obtained from patients who underwent surgery in the 253rd Hospital of PLA (Hohhot, Inner Mongolia, China) with signed informed consent. All fresh tissues samples were immediately frozen in liquid nitrogen and stored at −80°C until use. Pathological diagnosis of all tissues samples was confirmed by two independent pathologists. The Review Board of the 253rd Hospital of PLA reviewed and approved the present study.

### Cell culture and transfection

The human epidermal melanocyte HEMa-LP was obtained from Invitrogen (Carlsbad, U.S.A.) and cultured in Medium 254 and Human Melanocyte Growth Supplement-2 (Invitrogen). The human melanoma cell lines SK-MEL-2, SK-MEL-28, and A375 were obtained from American Type Culture Collection (ATCC). SK-MEL-2 and SK-MEL-28 cells were cultured in Eagle’s Minimum Essential Medium. A375 cells were cultured in Dulbecco’s Modified Eagle’s Medium. All cells were maintained in medium supplemented with 10% fetal bovine serum (Invitrogen) in an atmosphere containing 5% CO_2_ at 37°C.

miR-200a, miR-200b, and miR-429 inhibitors were obtained from GenePharma (Shanghai, China). All plasmids and miRNAs inhibitors were transfected using Lipofectamine 3000 (Invitrogen) following the manufacturer’s protocol.

### RNA extraction and quantitative real-time polymerase chain reaction (qRT-PCR)

Total RNA was isolated from tissues samples and cells using TRIzol (Invitrogen) following the manufacturer’s protocol. The RNA was treated with DNase I to remove genomic DNA. Reverse transcription was performed using the M-MLV Reverse Transcriptase (Invitrogen) following the manufacturer’s protocol. Quantitative real-time polymerase chain reaction (qRT-PCR) was performed on ABI StepOnePlus system (Applied Biosystems, Foster City, CA, U.S.A.). The expression of ILF3-AS1 was measured using SYBR® Premix Ex Taq™ II (Takara, Dalian, China) and normalized to GAPDH. The expression of miRNAs was measured using TaqMan MicroRNA Assays (Applied Biosystems) following the manufacturer’s protocol. The primer sequences used were as follows: 5′-TAAACCCCACTGTCTTCC-3′ (forward) and 5′-TTCCTTGCTCTTCTTGCTC-3′ (reverse) for ILF3-AS1; 5′-CTCTTGTGCCCCTTTCTT-3′ (forward) and 5′-ATGGCTTCTCGCATCCTAT-3′ (reverse) for HEIH; 5′-GGAGCGAGATCCCTCCAAAAT-3′ (forward) and 5′-GGCTGTTGTCATACTTCTCATGG-3′ (reverse) for GAPDH. The relative expression of RNAs was calculated using the comparative *C*_t_ method.

### Vectors and stable cell lines construction

Two independent cDNA oligonucleotides specifically targeting ILF3-AS1 (sh-ILF3-AS1-1 and sh-ILF3-AS1-2) were synthesized by GenePharma (Shanghai, China) and inserted into the shRNA expression vector pGPH1/Neo. The shRNAs target sites were as follows: for sh-ILF3-AS1-1: GCCTGTTGATTCAGACGTTCC; for sh-ILF3-AS1-2: GCTTTGTCCTTACAAGCGTGG. The shRNAs were transfected into A375 and SK-MEL-2 cells, and selected with neomycin (1000 µg/ml) for 4 weeks.

ILF3-AS1 full-length transcript was PCR amplified with the Phusion Flash High-Fidelity PCR Master Mix (Thermo Fisher, Waltham, MA, U.S.A.) and subcloned into the *Hin*d III and *Bam*H I sites of pcDNA3.1 (Invitrogen) or pSPT19 (Roche, Mannheim, Germany), named pcDNA3.1-ILF3-AS1 or pSPT19-ILF3-AS1 respectively. The primers used were as follows: 5′-CCCAAGCTTATCTTACGCCCGTCGCCCTGAG-3′ (forward) and 5′-CGGGATCCGACACGGGAAACAGGAGGATTTA-3′ (reverse). lncRNA HEIH overexpression vector pcDNA3.1-HEIH was constructed as previously described [31].

### Cell proliferation assays

Glo cell viability assays and ethynyl deoxyuridine (EdU) incorporation assays were performed to assess cell proliferation. For Glo cell viability assays, 3000 indicated melanoma cells were seeded in 96-well plates. The luminescence at each time point was acquired with the Cell Titer-Glo® Luminescent Cell Viability Assay (Promega, Madison, WI, U.S.A.) according to the manufacturer’s protocol. Cell viability was assessed using the proliferation curves plotted with the luminescence values. EdU incorporation assays were carried out using the EdU kit (Roche) according to the manufacturer’s protocol. The results were acquired and quantified using the Zeiss photomicroscope (Carl Zeiss, Oberkochen, Germany) and Image-Pro plus 6.0 software.

### Transwell migration and invasion assays

Transwell assays were carried out to assess cell migration and invasion capability. In brief, indicated melanoma cells were suspended in serum-free medium with 1 μg/ml Mitomycin C to inhibit cell proliferation, and seeded in the upper chamber of a 24-well transwell insert (8 μm pore size, Millipore, Bedford, MA, U.S.A.). For invasion assays, Coating Matrigel (BD Biosciences, San Jose, CA, U.S.A.) was plated in the upper chamber before the seeding of cells. The lower chamber was filled with complete medium. After being incubated for 24 h, the cells at the upper chamber were removed using cotton swabs, and the migratory or invasive cells at the bottom of the inserts were fixed by methanol, stained using Crystal Violet, photographed by Zeiss photomicroscope, and quantified by counting in five random fields.

### RNA pull-down assays

ILF3-AS1 and its antisense RNA were *in vitro* transcribed and biotin-labeled from vector pSPT19-ILF3-AS1 using the Biotin RNA Labeling Mix (Roche) and T7 or SP6 RNA polymerase (Roche) respectively. Then 50 pmol of biotin-labeled RNA was mixed with 1 mg of protein extracts from A375 cells for 1 h at 4°C, followed by being incubated with Dynabeads Myone Streptavidin T1 (Invitrogen) for additional 1 h. The proteins binding to the Dynabeads were resolved in SDS buffer and separated by sodium dodecyl sulfate/polyacrylamide gel electrophoresis, followed by being transferred to nitrocellulose membrane. Then the membranes were incubated with antibodies for EZH2 (Millipore) or GAPDH (Cell Signaling Technology, Boston, MA, U.S.A.). After being washed, the membranes were incubated with fluorescence-labeled secondary antibodies, and detected using an Odyssey infrared scanner (Li-Cor, Lincoln, NE, U.S.A.).

### RNA immunoprecipitation (RIP) assays

RNA immunoprecipitation (RIP) assays were performed using the EZ-Magna RIP™ RNA Binding Protein Immunoprecipitation Kit (Millipore) and EZH2 antibody (Millipore) following the manufacturer’s protocol. Retrieved RNA was reverse transcribed and measured by qRT-PCR as above described.

### Chromatin immunoprecipitation (ChIP) assays

Chromatin immunoprecipitation (ChIP) assays were performed using the EZ-Magna ChIP™ A/G Chromatin Immunoprecipitation Kit (Millipore) and EZH2 antibody (Millipore) or H3K27me3 antibody (Millipore) following the manufacturer’s protocol. Retrieved DNA was measured using SYBR® Premix Ex Taq™ II (Takara) on ABI StepOnePlus system (Applied Biosystems). The primer sequences were as follows: 5′-CTGCGTCACCGTCACTGG-3′ (forward) and 5′-ACAACTCGCCCGTCTCTG-3′ (reverse) for *miR-200b/a/429* promoter; 5′-GCTGGGCGTGACTGTTAC-3′ (forward) and 5′-GAGTGTGGTGTTGGGGGA-3′ (reverse) for *β-actin* promoter.

### Statistical analysis

Statistical analyses were implemented using the SPSS 18.0 software. Differences among the groups were estimated by Mann–Whitney *U* test, Log-rank test, Student’s *t* test, or Pearson’s correlation analysis as indicated. *P*<0.05 was considered as statistically significant.

## Results

### ILF3-AS1 is up-regulated in melanoma tissues and cell lines, and correlated with poor prognosis of melanoma patients

To investigate the expression of ILF3-AS1 in melanoma, we first searched the MiTranscriptome database (www.mitranscriptome.org) [8], and found that ILF3-AS1 is increased in primary melanomas and metastatic melanomas compared with normal human melanocytes (NHMEs) (Figure 1A). Furthermore, we collected 37 benign nevi, 60 primary melanomas, and 25 metastatic melanomas, and measured ILF3-AS1 expression by qRT-PCR. Our results showed that ILF3-AS1 is also significantly up-regulated in primary melanomas compared with benign nevi, and is further up-regulated in metastatic melanomas (Figure 1B). Analyzing the correlation between ILF3-AS1 expression and clinicopathological characteristics of these 60 primary melanomas, we noted that ILF3-AS1 is higher in melanomas at least 1 mm thick, which is more likely to metastasize and has more severity (T2/T3/T4 versus T1) (Figure 1C). To analyze the correlation between ILF3-AS1 expression and melanoma patients’ prognosis, we performed Kaplan–Meier survival analysis. As shown in Figure 1D, patients with higher ILF3-AS1 expression had a worse overall survival than those with lower ILF3-AS1 expression. These results showed that ILF3-AS1 is up-regulated in melanoma tissues and high ILF3-AS1 expression is correlated with metastatic characteristic and poor prognosis. Then we measured the expression of ILF3-AS1 in human epidermal melanocyte (HEMa-LP) and melanoma cell lines (SK-MEL-2, SK-MEL-28, and A375) by qRT-PCR. The results showed that ILF3-AS1 is significantly up-regulated in melanoma cell lines compared with epidermal melanocyte (Figure 1E).

**Figure 1:** ILF3-AS1 is up-regulated in melanoma tissues and cell lines, and indicates poor prognosis of melanoma patients (**A**) MiTranscriptome expression data for ILF3-AS1 across all available NHMEs (*n*=4), primary melanomas (*n*=33), and metastatic melanomas (*n*=228). (**B**) The expression of ILF3-AS1 in 37 benign nevi, 60 primary melanomas, and 25 metastatic melanomas was measured by qRT-PCR. (**C**) The expression of ILF3-AS1 in melanomas categorized based on tumor thickness at diagnosis. For (A)–(C), data are represented as median with interquartile range. *P* values were acquired by Mann–Whitney *U* test. (**D**) Kaplan–Meier survival analysis of the correlation between ILF3-AS1 expression and overall survival of melanoma patients. *P* values were acquired by log-rank test. (**E**) The expression of ILF3-AS1 in human epidermal melanocytes (HEMa-LP) and melanoma cell lines (SK-MEL-2, SK-MEL-28, and A375) was measured by qRT-PCR. Data are represented as mean ± SD; **P<0.01 by Student’s *t* test. (**F**) The expression of ILF3-AS1 in 13 breast tissues, 12 breast cancer tissues, and 8 metastatic breast cancer tissues was measured by qRT-PCR. (**G**) The expression of ILF3-AS1 in 11 lung tissues, 9 NSCLC tissues, and 6 metastatic NSCLC tissues was measured by qRT-PCR. For (F) and (G), data are represented as median with interquartile range. *P* values were acquired by Mann–Whitney *U* test.

To investigate the expression pattern of ILF3-AS1 in other tumors, we also collected 13 breast tissues, 12 breast cancer tissues, 8 metastatic breast cancer tissues, 11 lung tissues, 9 NSCLC tissues, and 6 metastatic NSCLC tissues. The results showed that ILF3-AS1 is also significantly up-regulated in breast cancer tissues and NSCLC tissues, compared with breast and lung tissues respectively (Figure 1F and G). Furthermore, ILF3-AS1 is also further up-regulated in metastatic breast cancer and NSCLC tissues (Figure 1F and G).

### Knockdown of ILF3-AS1 inhibits melanoma cell proliferation

To explore the biological function of ILF3-AS1 in melanoma cells, we stably depleted ILF3-AS1 in A375 cells using two independent ILF3-AS1 specific shRNAs (Figure 2A). Glo cell viability assays revealed that knockdown of ILF3-AS1 by both shRNAs significantly inhibits A375 cell proliferation (Figure 2B). EdU incorporation assays also revealed that knockdown of ILF3-AS1 in A375 cells significantly decreases percentage of EdU positive cells (Figure 2C). To further confirm the effects of ILF3-AS1 on melanoma cell proliferation, we stably depleted ILF3-AS1 in SK-MEL-2 cells using two independent ILF3-AS1 specific shRNAs (Figure 2D). Glo cell viability assays revealed that knockdown of ILF3-AS1 by both shRNAs significantly inhibits SK-MEL-2 cell proliferation (Figure 2E). EdU incorporation assays also revealed that knockdown of ILF3-AS1 in SK-MEL-2 cells significantly decreases percentage of EdU positive cells (Figure 2F). These results demonstrated that knockdown of ILF3-AS1 inhibits melanoma cell proliferation.

**Figure 2:** Knockdown of ILF3-AS1 inhibits melanoma cell proliferation (**A**) The expression of ILF3-AS1 in ILF3-AS1 stably depleted and control A375 cells. (**B**) Glo cell viability assays in ILF3-AS1 stably depleted and control A375 cells. (**C**) EdU incorporation assays in ILF3-AS1 stably depleted and control A375 cells. The blue color indicates the nuclei, and the red color indicates EdU-positive nuclei; scale bar = 100 μm. (**D**) The expression of ILF3-AS1 in ILF3-AS1 stably depleted and control SK-MEL-2 cells. (**E**) Glo cell viability assays in ILF3-AS1 stably depleted and control SK-MEL-2 cells. (**F**) EdU incorporation assays in ILF3-AS1 stably depleted and control SK-MEL-2 cells. The blue color indicates the nuclei, and the red color indicates EdU-positive nuclei; scale bar = 100 μm. For all panels, data are represented as mean ± SD; **P<0.01, ***P<0.001 by Student’s *t* test.

### Knockdown of ILF3-AS1 inhibits melanoma cell migration and invasion

To further explore the effects of ILF3-AS1 on melanoma cell migration and invasion, we performed transwell migration and invasion assays. The results revealed that the number of migrated A375 cells in ILF3-AS1 knockdown group is much fewer than that in the control group (Figure 3A). The number of invasive A375 cells in ILF3-AS1 knockdown group is also much fewer than that in the control group (Figure 3B). The effects of ILF3-AS1 on melanoma cell migration and invasion were further confirmed on SK-MEL-2 cells (Figure 3C and D). These results demonstrated that knockdown of ILF3-AS1 inhibits melanoma cell migration and invasion.

**Figure 3:** Knockdown of ILF3-AS1 inhibits melanoma cell migration and invasion (**A**) Transwell migration assays in ILF3-AS1 stably depleted and control A375 cells. Representative images are shown; scale bar = 100 μm. (**B**) Transwell invasion assays in ILF3-AS1 stably depleted and control A375 cells. Representative images are shown; scale bar = 100 μm. (**C**) Transwell migration assays in ILF3-AS1 stably depleted and control SK-MEL-2 cells. Representative images are shown; scale bar = 100 μm. (**D**) Transwell invasion assays in ILF3-AS1 stably depleted and control SK-MEL-2 cells. Representative images are shown; scale bar = 100 μm. For all panels, data are represented as mean ± SD; **P<0.01, ***P<0.001 by Student’s *t* test.

### ILF3-AS1 negatively regulates the expression of miR-200b/a/429 via binding to EZH2

Increasing evidence have revealed that many lncRNAs bind and recruit EZH2 to target genes [32,33]. EZH2 is an important subunit of polycomb repressive complex 2 (PRC2), which increases H3K27me3 levels across the promoters of target genes and inhibits the expression of target genes [34]. To test whether ILF3-AS1 also functions in such a manner, we performed RNA pull-down assays using *in vitro* transcribed biotin-labeled ILF3-AS1. The results showed that ILF3-AS1 specifically binds to EZH2, but not GAPDH protein (Figure 4A). To further confirm the interaction between ILF3-AS1 and EZH2, RIP assays with EZH2 specific antibody were performed. As shown in Figure 4B, a significant enrichment of ILF3-AS1, but not GAPDH mRNA with EZH2 antibody was observed. lncRNA HEIH was used as positive control, which has been reported to associate with EZH2 [35]. miR-200b/a/429 is a well-known EZH2 target gene [36], which also has crucial roles in the proliferation, migration, and invasion of melanoma cells. To investigate whether ILF3-AS1 is involved in the transcriptional regulation of miR-200b/a/429 via interacting with EZH2, we performed ChIP assays using EZH2 and H3K27me3 specific antibodies in ILF3-AS1 stably depleted and control A375 cells. As shown in Figure 4C, knockdown of ILF3-AS1 decreased the binding of EZH2 and H3K27me3 levels across the *miR-200b/a/429* promoter, but not the *β-actin* promoter. Furthermore, knockdown of ILF3-AS1 up-regulates miR-200b/a/429 expression in both A375 cells and SK-MEL-2 cells (Figure 4D and E). Collectively, these results demonstrated that ILF3-AS1 binds to EZH2, recruits EZH2 to the *miR-200b/a/429* promoter, up-regulates H3K27me3 levels across the promoter, and represses the expression of miR-200b/a/429.

**Figure 4:** ILF3-AS1 negatively regulates miR-200b/a/429 expression via interacting with EZH2 (**A**) RNA pull-down assays followed by Western blot analysis revealed the specific enrichment of EZH2, but not GAPDH protein with *in vitro* transcribed biotin-labeled ILF3-AS1 compared with antisense RNA (negative control). (**B**) RIP assays followed by qRT-PCR revealed the specific enrichment of ILF3-AS1, but not GAPDH mRNA with EZH2 antibody compared with nonspecific IgG (negative control). HEIH was used as positive control. (**C**) The specific binding of EZH2 and H3K27me3 levels across the *miR-200b/a/429* promoter and the *β-actin* promoter in ILF3-AS1 stably depleted and control A375 cells were measured by ChIP assays followed by qPCR. (**D**) The expression of miR-200b, miR-200a, and miR-429 in ILF3-AS1 stably depleted and control A375 cells was measured by qRT-PCR. (**E**) The expression of miR-200b, miR-200a, and miR-429 in ILF3-AS1 stably depleted and control SK-MEL-2 cells was measured by qRT-PCR. Data are represented as mean ± SD; *P<0.05, **P<0.01, ***P<0.001 by Student’s *t* test.

### The expression of ILF3-AS1 is negatively correlated with that of miR-200b/a/429 in melanoma tissues

To explore whether the regulation of miR-200b/a/429 by ILF3-AS1 also exists *in vivo*, we measured the correlation between the expression of ILF3-AS1 and miR-200b/a/429 in melanoma tissues. The results showed that the expression of ILF3-AS1 is negatively correlated with that of miR-200b, miR-200a, and miR-429 in melanoma tissues (Figure 5A–C), supporting the regulation of miR-200b/a/429 by ILF3-AS1 *in vivo*.

**Figure 5:** The correlation between ILF3-AS1 and miR-200s expression in melanoma tissues The correlation between ILF3-AS1 expression level andmiR-200b (**A**), miR-200a (**B**), and miR-429 (**C**) expression levels in 60 melanoma tissues. *P* values were acquired by Pearson’s correlation analysis.

### Inhibition of miR-200b/a/429 abrogates the repressing effects of proliferation, migration, and invasion caused by ILF3-AS1 knockdown

To explore whether the regulation of miR-200b/a/429 mediates the biological effects of ILF3-AS1 on melanoma cell proliferation, migration, and invasion, we inhibited miR-200b/a/429 expression by transfecting miR-200b/a/429 inhibitors in ILF3-AS1 stably depleted A375 cells (Figure 6A). Glo cell viability assays and EdU incorporation assays revealed that inhibition of miR-200b/a/429 abrogates the proliferation repression caused by ILF3-AS1 knockdown (Figure 6B and C). Furthermore, transwell migration and invasion assays revealed that inhibition of miR-200b/a/429 abrogates the migration and invasion repression caused by ILF3-AS1 knockdown (Figure 6D and E). These results demonstrated that the repressing effects of proliferation, migration, and invasion caused by ILF3-AS1 knockdown are dependent on miR-200b/a/429.

**Figure 6:** Inhibition of miR-200b/a/429 abrogates the inhibitory effects of ILF3-AS1 knockdown on melanoma cell proliferation, migration, and invasion (**A**) The expression of miR-200b, miR-200a, and miR-429 in ILF3-AS1 stably depleted and control A375 cells transfected with miR-200b/a/429 inhibitors or control was measured by qRT-PCR. (**B**) Glo cell viability assays in ILF3-AS1 stably depleted and control A375 cells transfected with miR-200b/a/429 inhibitors or control. (**C**) EdU incorporation assays in ILF3-AS1 stably depleted and control A375 cells transfected with miR-200b/a/429 inhibitors or control. The blue color indicates the nuclei, and the red color indicates EdU-positive nuclei; scale bar = 100 μm. (**D**) Transwell migration assays in ILF3-AS1 stably depleted and control A375 cells transfected with miR-200b/a/429 inhibitors or control. Representative images are shown; scale bar = 100 μm. (**E**) Transwell invasion assays in ILF3-AS1 stably depleted and control A375 cells transfected with miR-200b/a/429 inhibitors or control. Representative images are shown; scale bar = 100 μm. For all panels, data are represented as mean ± SD; **P<0.01, ***P<0.001 by Student’s *t* test.

### Enhanced expression of ILF3-AS1 promotes melanoma cell proliferation and invasion

A previous report showed that lncRNA HEIH also has oncogenic roles in melanoma via repressing miR-200b/a/429, which is consistent with the action mechanisms of ILF3-AS1 in melanoma. Therefore, we next investigated whether the oncogenic role of ILF3-AS1 is redundant with that of HEIH in melanoma. Glo cell viability assays revealed that enhanced expression of ILF3-AS1 significantly promotes A375 cell proliferation, and concurrent overexpression of ILF3-AS1 and HEIH slightly further promotes A375 cell proliferation (Figure 7A). Transwell invasion assays revealed that enhanced expression of ILF3-AS1 significantly promotes A375 cell invasion, and concurrent overexpression of ILF3-AS1 and HEIH slightly further promotes A375 cell invasion (Figure 7B). These results demonstrated that overexpression of ILF3-AS1 promotes melanoma cell proliferation and invasion, which is at least partially redundant with the roles of HEIH in melanoma.

**Figure 7:** Overexpression of ILF3-AS1 promotes melanoma cell proliferation and invasion, which is partially redundant with the roles of HEIH in melanoma (**A**) After transient transfection of ILF3-AS1 overexpression plasmids or cotransfection of ILF3-AS1 and HEIH overexpression plasmids into A375 cells, Glo cell viability assays were performed in these cells. (**B**) After transient transfection of ILF3-AS1 overexpression plasmids or cotransfection of ILF3-AS1 and HEIH overexpression plasmids into A375 cells, transwell invasion assays were performed in these cells; **P<0.01 by Student’s *t* test.

## Discussion

As one of the deadliest skin cancer, the incidence of melanoma is increasing faster than most of other solid cancers worldwide [37]. The tumorigenesis and progression of melanoma involve complex changes in many genes networks [38]. Among the critical molecules involved in the pathogenesis of melanoma, lncRNAs gradually attract human’s attentions for their important roles in melanoma [39]. For example, lncRNA SLNCR1 associates with poor melanoma survival and increases melanoma invasion via transcriptionally activating MMP9 [30]. SAMMSON functions as an oncogene in melanoma and silencing SAMMSON delivers effective antimelanoma therapeutic responses [12]. MALAT1 promotes melanoma growth and metastasis via sponging miR-22 [40]. BANCR promotes melanoma proliferation via activating MAPK pathway [41]. Also in our previous study, we found that MHENCR promotes melanoma growth and metastasis via activating PI3K–Akt pathway [42]. In our another previous report, we found that PVT1 is up-regulated in melanoma tissues and serum of melanoma patients. Functional experiments demonstrated that PVT1 promotes melanoma cell proliferation and migration. These evidence further confirm the critical roles of lncRNAs in melanoma. The amount of lncRNAs is much larger than that of protein-coding mRNAs [8], and many genes are involved in melanoma [43]. Thus, it is important to further reveal more functional lncRNAs in melanoma.

Searching the differently expressed lncRNAs in a previously reported RNA sequencing results of melanoma [30], we noted a novel lncRNA ILF3-AS1, which localizes at chromosome 19p13.2 and is up-regulated in melanoma tissues. The MiTranscriptome database also demonstrates that ILF3-AS1 is up-regulated in melanoma. However, the functions of ILF3-AS1 in cancers are unknown. In the present study, we further examined the expression, clinical significances, and biological roles of ILF3-AS1 in melanoma. We found that ILF3-AS1 is up-regulated in melanoma tissues and cell lines, and associates with metastatic characteristic and poor prognosis of melanoma patients. Functional assays demonstrated that silencing of ILF3-AS1 using two independent shRNAs both significantly inhibit melanoma cell proliferation, migration, and invasion. Overexpression of ILF3-AS1 promotes melanoma cell proliferation and invasion. These data reveal that as a previously unknown lncRNA, ILF3-AS1 is dysregulated and also has critical functions in melanoma. Our study enlarges our recognitions of lncRNAs and provides a novel prognostic biomarker and therapeutic target for melanoma.

miR-200s is known to have complex roles in many cancer processes, including proliferation, migration, invasion, drug resistance, epithelial–mesenchymal transition, and et al. [44–46]. miR-200s has also been reported to be down-regulated in invasive melanoma [28]. But the factors contributing to miR-200s dysregulation in melanoma are still unknown. In the present study, we found that ILF3-AS1 interacts with EZH2. EZH2 is a histone methyltransferase, catalyzes H3K27 trimethylation, and inhibits target genes expression. In the present study, we further found that through interacting with EZH2, ILF3-AS1 recruits EZH2 to the *miR-200b/a/429* promoter, up-regulates H3K27me3 levels across the *miR-200b/a/429* promoter, and inhibits miR-200b/a/429 expression. The expression of ILF3-AS1 is negatively correlated with that of miR-200b/a/429 in melanoma tissues. Silencing miR-200b/a/429 abrogates the repressive effects of ILF3-AS1 knockdown on melanoma cell proliferation, migration, and invasion. These data demonstrate that ILF3-AS1 epigenetically silences miR-200b/a/429 expression and the biological roles of ILF3-AS1 in melanoma are dependent on miR-200b/a/429.

In conclusion, our results identify a previously unknown lncRNA ILF3-AS1, which is up-regulated in melanoma, associates with poor prognosis of melanoma patients, and promotes melanoma cell proliferation, migration, and invasion. Mechanistically, ILF3-AS1 interacts with EZH2 and epigenetically silences miR-200b/a/429. Our data imply that ILF3-AS1 would be a potential prognostic biomarker and therapeutic target for melanoma.

## Abbreviations

ChIP: chromatin immunoprecipitation
Edu: ethynyl deoxyuridine
ILF3-AS1: ILF3 antisense transcript 1
lncRNA: long noncoding RNA
NHME: normal human melanocyte
NSCLC: non-small cell lung cancer
PRC2: polycomb repressive complex 2
qRT-PCR: quantitative real-time polymerase chain reaction
RIP: RNA immunoprecipitation
